# Effects of exercise and psychological interventions on smartphone addiction among university students: A systematic review

**DOI:** 10.3389/fpsyg.2022.1021285

**Published:** 2022-10-05

**Authors:** Huange Liu, Kim Geok Soh, Shamsulariffin Samsudin, Watnawat Rattanakoses, Fengmeng Qi

**Affiliations:** ^1^Department of Sports Studies, Faculty of Educational Studies, Universiti Putra Malaysia, Seri Kembangan, Malaysia; ^2^Department of Khon Kaen Sport School, Thailand National Sports University, Bueng Nam Rak, Thailand

**Keywords:** exercise, psychological, intervention, smartphone addiction, university students

## Abstract

**Background and aims:**

Among the large number of studies on smartphone addiction, only a few randomized controlled trials on exercise and psychological interventions for smartphone addiction by university students have been published. This study aims to systematically investigate the impact of exercise and psychological interventions on smartphone addiction among university students.

**Methods:**

The PRISMA guidelines were adopted for this systematic literature review. Prominent academic databases such as Web of Science, PubMed, ProQuest, Cochrane Library, China National Knowledge Infrastructure (CNKI) and PsycINFO were searched to find eligible studies published before Aug 2021. The overall quality of the articles was checked using the “QualSyst” tool by Kmet et al.

**Results:**

From among 600 papers, 23 met the inclusion criteria and were incorporated into our systematic review. All of the studies were randomized controlled trials. The following thematic areas emerged as a result of the content analysis: study selection and design, as well as study characteristics (participants, intervention, comparisons, and outcomes).

**Discussion and conclusion:**

The literature on exercise and psychological interventions for smartphone addiction is scarce. There is a need to introduce new interventions and to validate the effectiveness of combined interventions. Our findings suggest that exercise and psychological interventions may help to reduce smartphone addiction. This combination was more effective compare to exercise or psychological intervention on mental health and addiction among university students. Future research should combine exercise and psychological interventions, focusing on university students, especially females, who are vulnerable to smartphone addiction. Further studies should focus on the cross-section of neuropsychology, cognitive psychology, and sports science to provide combined interventions in physiological and psychological direction.

**Systematic review registration:**

https://www.crd.york.ac.uk/prospero, identifier: CRD42021278037.

## Introduction

Mobile-based technology is advancing at an unprecedented rate, and in the past decade, the amount of smartphone users has increased substantially on a global scale. Smartphones offer people with a convenient and practical approaches to enrich their social lives (Sahu et al., 2019; Lu et al., 2020). But even though they offer many advantages, smartphone use issues have slowly started to become a major health concern (Billieux, 2012; Elhai et al., 2017; Lu et al., 2020).

Smartphone addiction (SA) is the theoretical defined criteria of behavioral addiction, which include the psychological (craving, cognitive salience, loss of control, and mood modification), physical dependence (tolerance and withdrawal symptoms), saliency, impulsivity, spotlight behavior, and relapse (Griffiths, 1995, 2005; Yen et al., 2009; Billieux et al., 2015; Panova and Carbonell, 2018). Smartphone addiction core signs and symptoms consist of obsessive thoughts about mobile telephones (craving), spending extra time on smartphones (tolerance), and experiencing anxiousness when smartphone is unavailable (withdrawal) (Kim et al., 2015; Peng et al., 2021).

Smartphone addiction comprises four properties: compulsion, withdrawal, and tolerance, and functional Impairment (Lin et al., 2014; Cha and Seo, 2018; Wang et al., 2018). Smartphone addiction is typically characterized by a feeling of anxiety (Bian and Leung, 2014; Gutiérrez et al., 2016; Shoukat, 2019), impaired attention (Wacks and Weinstein, 2021), impaired function (Lin et al., 2014; Matar Boumosleh and Jaalouk, 2017; Mehrnaz et al., 2018; Alageel et al., 2021), and reduced decision-making ability.

The maintenance of the psychological underpinnings of smartphone addiction remains to be unknown (Mehmood et al., 2021). Predisposing factors, cognitive responses to external and internal stimuli, executive functionality (e.g., decision-making behavior and inhibitory control) are all taken into consideration by the I-PACE model (Mehmood et al., 2021). The addiction to mobile phones is a unique behavioral addiction issue whereby a person's physical, social, and psychological are impaired, and this leads to harmful social consequences (Billieux et al., 2015; Mehrnaz et al., 2018). Prior work has mentioned that loss of control (e.g., affected decision-making processes and decreased impulse control) is a major issue due to smartphone addiction (Billieux, 2012; Billieux et al., 2015). Based on the available literature, impulsivity is a lead cause of addictive behavior (Groman et al., 2009; Weafer et al., 2014; Billieux et al., 2015). Smartphone addiction has inevitably become a significant health issue among university students with poorer mental health (Ding et al., 2021). Excessive smartphone use can lead to severe distractions (Liu et al., 2019). The development of technology not only brings convenience to the study and life of university students, but also may bring negative consequences (Lu et al., 2020). Difficult academic homework and concern about the future may contribute to university students' high levels of stress; students are more inclined to turn to use their phones for reducing stress when confronted with these challenges (Gazzaz et al., 2018; Mehmood et al., 2021). To use a smartphone in a stressful situation, according to Beranuy et al. (2009), it could be regarded as a type of alternative satisfaction, or as a form of addiction (Beranuy et al., 2009; Mehmood et al., 2021). Students are more probable to become addicted to smartphones if they are more stressed (Mehmood et al., 2021). According to the general strain theory, strains or stressors increase the probability of negative emotions like anger and frustration, thus leading to corrective behavior (Jun and Choi, 2015; Mehmood et al., 2021). However, engaging in smartphone addiction behavior might be a method of reducing stress or manage with negative emotions. Several research have shown that students are more probable to become addicted to smartphones if they are more stressed (Mehmood et al., 2021).

There exists substantial evidence that vulnerable people with poor self-control can become more addicted to smartphone misuse. The use and gratifications theory (Ruggiero, 2009) enlightens us that the forming process of mobile phone dependence may include the psychological needs of college students who rely on mobile phones to use them much more frequently. Although the psychological needs of university students addicted to mobile phones are different from each other, they all lead to the same result: they are addicted to mobile phone use and cannot extricate themselves. University students who have an addiction to smartphones are characterized as becoming bored quickly, and have a low response inhibition, poor planning skills, and the tendency to feel lost without their smartphone (Panza et al., 2019; Pengpid and Peltzer, 2019; Ding et al., 2021).

Since the last decade, smartphone addiction with today's children and young people (CYP) has been one of the major global health problems (Sohn et al., 2019). Smartphone addiction has significantly afflicted university students' physical and intellectual fitness, and related reports point out that cellular smartphone addiction has turned out to be a label of university students. According to a survey conducted in China in 2016, 21.3% of university students were addicted to their smartphones (Long et al., 2016; Mehmood et al., 2021). Furthermore, according to a survey conducted in South Korea in 2013, 25% of university students are at a great risk of becoming dependent on their smartphones (Jun, 2016; Mehmood et al., 2021). Therefore, the issue of student smartphone addiction has already attracted much attention.

Previous studies have shown that smartphone use is negatively correlated with the intensity of exercise. Systematic physical activity can effectively alleviate smartphone addiction (mainly behavioral and adjuvant therapies) (Kim, 2013). However, evidence-based interventions regarding smartphone addiction behavior among university students are lacking. The main intervention measures for smartphone addiction include group psychological counseling, mindfulness intervention (Li et al., 2017b; Garland and Howard, 2018; Lan et al., 2018; Sancho et al., 2018), meditation (Choi et al., 2020) and cognitive behavior therapy (Kim et al., 2012; Ajay Krishna et al., 2014; Zhang Y. Y. et al., 2020; Singh and Samantaray, 2021).

Previous research has proven that exercise interventions can fix and alter rather excited nerve cells and beautify their adaptability to external modifications (Kim, 2013; Tang and Lee, 2021). Exercise has been shown to reduce smartphone addiction by university students (Kai, 2016; Xingtong and Chao, 2016; Fan et al., 2021). However, there is a lack of comprehensive intervention measures combining exercise and psychological intervention, especially as an emerging combined intervention method. Exercise and psychological intervention in college students' mobile phone addiction merits further research to provide empirical evidence.

Previous systematic reviews have focused on exercise as an alternative to treat smartphone addiction. The results indicate that exercise interventions have a positive effect on the treatment of smartphone addiction, with longer intervention times associated with better intervention outcomes. There is evidence in the literature that a combination of exercise and psychological interventions effectively overcome problematic smartphone use among university students, reducing smartphone addiction, loneliness, anxiety, and stress levels. However, there is a lack of related research combining exercise and psychological intervention. Therefore, this review aims to investigate the evidence obtained on the effects of exercise or psychological interventions to smartphone addiction.

The objective of this research is to use RCTs that examine the impact and effectiveness of a smartphone ad-diction intervention based on exercise and psychology. The hypothesis of this study was that smartphone addiction universities that participated in combined exercise and psychological interventions were better able to reduce addiction than university students who participated in exercise or psychological interventions. This review is necessary because of the lack of systematic review focused on combining exercise with psychological intervention.

## Methods

The Preferred Reporting Items for Systematic Reviews and Meta-Analyses (or PRISMA) statement was utilized in reporting this review (Moher et al., 2009). The a priori procedure used was released by the PROSPERO international prospective registrar of systematic reviews (https://www.crd.york.ac.uk/prospero), CRD42021278037.

### Search resources methods

Two reviewers performed the literature retrieval, using various prominent database sources such as PubMed, Cochrane Library, Web of Science, ProQuest, China National Knowledge Infrastructure (CNKI), and PsycINFO citations and references, as well as gray literature, from inception, to August 2021. The bibliography lists of all RCTs included in the study were manually retrieved, limiting the search procedure to papers published in the title, abstract, or keywords, and limited to the English and Chinese languages.

The search was carried out on the 29th of August, 2021. A search was performed by title or abstract for each of the databases. The search strategy used a predefined combination of MESH terms and keywords: ([Title/Abstract] (“Internet Addiction Disorder”[Mesh] OR Addiction Disorder^*^, Internet OR Disorder^*^, Internet Addiction OR “Internet Addiction Disorder^*^ OR” Internet Addiction^*^ OR Addiction^*^, Internet OR “Social Media Addiction^*^” OR Addiction^*^, Social Media OR Media Addiction^*^, Social OR Addiction^*^, Smartphone OR “Internet Gaming Disorder^*^” OR Disorder^*^, Internet Gaming OR Gaming Disorder^*^, Internet OR “Mobile Phone Addiction OR “Mobile Phone Addiction Tendency” OR “Smartphone Overuse OR “Mobile Phone Overuse” OR “Problematic Smartphone Use” OR “Excessive Mobile Phone Use” OR “Problematic Cell Phone Use”) AND([Title/Abstract] (“Exercise”[Mesh] OR “Exercise^*^” OR “Physical Activity^*^” OR Activit^*^, Physical OR Exercise^*^, Physical OR “Physical Exercise^*^” OR “Acute Exercise^*^” OR Exercise^*^, Acute OR Exercise^*^, Isometric OR “Isometric Exercise^*^” OR Exercise^*^, Aerobic OR “Aerobic Exercise^*^” OR “Exercise Training^*^” OR Training^*^, Exercise OR “Sport^*^” OR “Football” OR “Basketball” OR “Baduanjin” OR “Mind-Body Exercise” OR “Tai Chi OR “Yoga” OR “Badminton” OR “Volleyball” OR “Run” OR “Outdoor Games OR “Psychosocial Intervention” OR Psychosocial Intervention^*^ OR Intervention^*^, Psychosocial OR Intervention^*^, Psychological OR Group Counseling Programs OR group psychotherapy OR Psychotherapy, Group OR Therapy, Group OR Group Therapy OR Mindfulness OR Cognitive Behavioral Therapy) AND ([Title/Abstract] (“Randomized Controlled Trial” OR “Randomized Controlled Trials as Topic” OR “Controlled Clinical Trial” OR randomized controlled trial OR randomized OR randomly OR trial). The same Chinese version of the English keywords were used for the CNKI database.

### Eligibility criteria

In this study, the standards for document retrieval, inclusion, screening, and exclusion were established based on strict adherence to the PRISMA statement and five specifications including P (i.e., Population), I (i.e., Intervention), C (i.e., Comparison), O (i.e., Outcome), and S (i.e., Study Design) (Liberati et al., 2009). The eligibility criteria for the considered studies were defined as follows. The study should include: (1) participants in the primary research who were university students and described as mobile phone dependent/addicted; (2) the primary interventions in the experimental group are exercise and psychological intervention.; (3) it was a sequence of RCTs; (4) employed a pre/posttest framework; (5) at least one result was reported (all result measures are available in Section Study selection). The exclusion criteria considered were as follows: (1) repeatedly published documents; (2) literature reviews as well as meta-analyses; (3) descriptive studies or case-control studies; (4) quasi-experimental studies, (5) qualitative reports; (6) case reports; (7) papers with only abstract but no full text; (8) non-randomized controlled research designs such as self-controlled experiments; (9) studies with no control group; and (10) papers with incomplete or incorrect outcome data.

### Study selection

The studies considered were added into EndNoteX9 reference management software to remove duplicates. Two researchers (i.e., HL, FQ) individually reviewed the studies that were initially added based on the inclusion criteria. When the researchers disagreed, a third reviewer (i.e., KS) checked the study to reach an agreement.

### Data extraction

The researchers individually searched the literature and extracted relevant data. After the screening and extraction of data, cross-checking into the analysis process; the final selection of the articles was determined by reaching an agreement by both reviewers. The predetermined population, intervention, control, and outcomes (PICO) criteria format was followed (Moyer, 2008). General information extracted by the reviewers included: (1) Author, title, publication year; (2) Details of the participants (age, gender, level of smartphone addiction); (3) Intervention type (type, duration, frequency, week; experimental group size, control group size, gender, intervention measures of the experimental group, intervention measures of the control group, evaluation tools of outcome indicators vs. non- exercise and psychological interventions, or vs. no treatment; (4) Type of outcome measure (validated scales for measuring and related results); and (5) Length of follow-up sessions. One author placed the information into a standard table, and the other author checked and confirmed it.

### Outcome measures

The outcome measures include primary outcome variables, secondary outcome variables and other variables used in the study, especially those designed to assess the effect of the intervention, including specific measurement variables (such as questionnaire scale results, physiological measures).

The primary outcome measured in this systematic review were the difference among exercise and psychological intervention in decreasing symptoms associated of smartphone addiction. Integrating the impact of different scales measuring symptoms related to smartphone addiction (such as MPAI, MPATS, SAS-C), it needs to be based on the theoretical definition and properties of smartphone addiction. Smartphone addiction is usually measured using subjects' self-reported questionnaires. It is characterized by continuous variables. Different smartphone addiction scales have different scoring criteria. For example, the Mobile Phone Addiction Index (MPAI) scores above 40 (Lu et al., 2020; Xiao et al., 2021), Smartphone Addiction Scale (SAS-C) score of 4 or above (Kai, 2016), Mobile Phone Addiction Tendency Scale for College Students (MPATS) scores above 48 were considered to smartphone addiction (Fan et al., 2021).

In addition, the primary outcome measure usually used in RCT studies of psychological interventions are evaluations/measures of mental health (such as depressive symptoms, anxiety symptoms). The main outcomes in this systematic review additionally include Emotional vs. Social Loneliness (ESLS), Sleep Quality, Cognitive Emotion Regulation (CERQ- C), Social Avoidance and Distress (SAD), and Wellbeing, quality of life (QOL), anxiety, loneliness.

The secondary outcome measured were loneliness, stress, and Field's Feelings of Inadequacy. Furthermore, include the follow-up.

### Quality assessment

Evaluation of the quality of the research reviewed for inclusion in the report was investigated by the quantitative assessment tool referred to as “QualSyst” (Kmet et al., 2004). The internal effectiveness of research or design, implementation, and analysis were used to minimize the degree of errors and deviations, which comprise 14 items (**Table 3**). The score was based on the level the specific criteria satisfied (i.e., no = 0, partial = 1, yes = 2). The letter “NA” represents items that do not apply to the study framework and were discarded from the computation of the overall summary score, The scores representing low, medium and high quality are ≤ 55%,55–75%, ≥75%; any low-quality study should be excluded from the systematic review (Kmet et al., 2004).

## Results

### Study design and selection

The primary search resulted in 600 individual articles, as shown in the flow chart in Figure 1. Using the PRISMA format requirements, 87 full-text studies were checked for eligibility by removing duplicative and screening records. A total of 36 were discarded (e.g., qualitative synthesis, did not provide a correlation table or statistics that can be transformed to correlations). A total of 51 articles were reports assessed for eligibility, of which 28 articles were discarded (e.g., not university students, no relevant intervention, non-randomized controlled study design, no relation with smartphone addiction, or not quality research). Finally, 23 papers satisfied the inclusion and narrative synthesis criteria (see Appendices S1, S2). The 23 papers that were considered were RCTs published in either English or Chinese (Figure 1). The quality of these tests was assessed (Table 1).

**Figure 1:** PRISMA flow chart of the study selection process.

**Table 1:** Quality assessment “QualSyst”.

**References **	**Question/** **objectivedescribed **	**Appropriate Study design **	**Appropriate** **subjectselection**	**Characteristics sufficiently described **	**Random allocation **	**Researchersblinded **	**Subjects blinded **	**Outcome measures well defined and robust to bias **	**Appropriate samplesize**	**Analytic methodswell described**	**Estimate of variance reported **	**Controlled for confounding **	**Results reported indetail**	**Conclusion supported by results? **	**Rating **
Renkai et al. (2015)	2	2	2	2	1	0	1	2	2	2	2	1	2	2	High
Lirong (2015)	2	2	2	2	1	0	0	2	1	2	2	0	2	2	Medium
Xingtong and Chao (2016)	2	2	2	0	NA	0	1	2	2	2	1	1	1	2	Medium
Rongchang and Xiaoyang (2015)	2	2	0	0	NA	0	0	2	2	2	1	0	0	1	Medium
Kai (2016)	2	2	2	2	2	0	0	2	2	2	1	1	2	2	High
Jingsong et al. (2016)	2	2	2	2	2	1	1	2	2	2	2	0	2	2	High
Ganfang (2017)	2	2	2	2	2	0	0	2	2	2	2	1	2	1	High
Xiaoni et al. (2019)	2	2	2	2	1	0	0	2	2	2	2	1	2	2	High
Xiao et al. (2021)	2	2	2	2	2	2	2	2	2	2	2	2	2	2	High
Fan et al. (2021)	2	2	2	2	2	2	2	2	1	2	2	2	2	2	High
Yu and Fumin (2007)	2	2	2	1	0	0	0	2	2	2	1	NA	2	2	Medium
Weifang et al. (2007)	2	2	2	2	1	0	0	2	2	2	2	1	2	2	High
Wenhai and Jiamei (2009)	2	2	2	2	1	0	0	2	2	2	2	1	1	2	High
Wei et al. (2010)	2	2	2	2	1	0	1	2	2	2	2	1	2	2	High
Ming et al. (2011)	2	2	2	2	1	0	0	2	2	2	2	0	2	2	High
Li et al. (2017a)	2	2	2	2	1	0	1	2	2	2	2	1	1	2	High
Rui et al. (2018)	2	2	2	1	1	0	0	2	2	2	2	1	2	1	Medium
Lan et al. (2018)	2	2	2	2	1	0	0	2	1	2	2	0	2	2	Medium
Zaihua et al. (2019)	2	2	1	1	1	0	0	2	2	2	2	0	1	2	Medium
Zhang X. et al. (2020)	2	2	2	2	1	0	0	2	1	2	2	0	2	1	Medium
Alavi et al. (2021)	2	2	2	2	1	0	0	2	2	2	2	2	2	2	High
Lu et al. (2020)	2	2	2	2	2	1	2	2	2	2	2	2	2	2	High
Yuxia et al. (2021)	2	2	2	2	2	0	0	2	2	2	2	2	2	2	High

NA, not applicable, 2 indicates yes, 1 indicates partial, 0 indicates no Quality; Quality score: ≥ 75% high, 55–75% medium, ≤ 55% low.

**Calculate the summary score:** Total sum = (number of “yes” ^*^ 2) + (number of “partials” ^*^ 1); Total possible sum = 28 – (number of “N/A” ^*^ 2).

**Summary score:** total sum/total possible sum.

### Study characteristics

#### Participants

The considered studies reported 2,215 participants. The average age of the participants was 19.65 ± 1.64, and the age range was 18–23. This was obtained from 23 studies. From among them, 22 involved both males and females. One study included only female data (Xiaoni et al., 2019). Additionally, the population of two studies involved freshmen (Lirong, 2015; Rongchang and Xiaoyang, 2015) and of one study were first- and second-year students (Yuxia et al., 2021), The target population of 15 studies was focused on individuals with a mild-to-moderate level of smartphone addiction, three studies focused on smartphone addiction of severe level. However, five studies did not report the inclusion criteria for smartphone addiction in the target population. The most prominent inclusion criteria were as follows:

1. Age ≥ 18 years (male or female).
2. Good health, no apparent speech disorder (Ming et al., 2011).
3. Diagnosed as an internet addict based on internet addiction test (or IAT), meeting diagnostic criteria for SA.
4. IAD (Smartphone Addiction and Internet Addiction Disorder) (Alavi et al., 2021).
5. Freshmen, sophomores, and third year of college.
6. No participation in similar research projects before (using medication for psychiatric problems and undergoing other psychotherapeutic remedies) (Alavi et al., 2021).
7. With no cardiovascular, renal metabolic, or pulmonary diseases, psychological disorders, or a history of alcohol abuse (Lu et al., 2020).
8. No regular exercise or psychotherapy in the past 6 months (Fan et al., 2021).
9. Have time to ensure that you can attend every counseling on time.
10. Smartphone addiction level was mild-to-moderate (40–60 points).
11. Agreed to be randomized.

Several RCTs demonstrated different inclusion criteria, which were as follows:

(1) 17–21 (Wenhai and Jiamei, 2009), 17–23 (Rui et al., 2018).
(2) University students with severe level of smartphone addiction (Lirong, 2015; Renkai et al., 2015; Lan et al., 2018).
(3) Two studies do not report mean age or age range (Ming et al., 2011; Zaihua et al., 2019).
(4) Students self-reported using the mobile internet for more than 6 h per day and the duration was ≥3 months (Yuxia et al., 2021).
(5) They did no longer take part in any standard exercise (e.g., running, walking, weight training, etc.) in the previous 3 months (Lu et al., 2020).
(6) Seven studies did not report smartphone addiction level (Wenhai and Jiamei, 2009; Ming et al., 2011; Rongchang and Xiaoyang, 2015; Rui et al., 2018; Zaihua et al., 2019; Alavi et al., 2021).

The primary exclusion criteria were as follows:

According to the exercise training intervention requirement, they must be able to move independently without any assisting device (Lu et al., 2020).

1) They had no significant disease (respiratory illness, musculoskeletal disorder, dementia and metabolic, cardiovascular disease, and renal or pulmonary diseases) that can affect them to participate in exercise or psychological treatment (Fan et al., 2021; Xiao et al., 2021);
2) Normal or corrected vision, without color blindness or weakness (Fan et al., 2021);
3) They were not diagnosed with psychosis or any severe psychiatric disorders (e.g., including other addictive disorders such as bipolar, personality, or antisocial personality, eating, obsessive-compulsive, or posttraumatic stress disorder) or attention disorders (Alavi et al., 2021);
4) The suicide risk was low.
5) Those who are unable to move due to injury or illness and drop out of school (Rui et al., 2018);
6) Those who were undergoing other psychotherapeutic treatments were also excluded from the study (Alavi et al., 2021).

The exclusion criteria were as follows:

1. Excluded students who scored below 47 on the Mobile Phone Addiction Tendency Scale for university students (MPATS) (Fan et al., 2021).
2. Mobile Phone Addiction Index (MPAI) scores below 40 (Lu et al., 2020; Xiao et al., 2021).
3. Excluded students who scored below 40 on the Mobile Phone Addiction Tendency Scale (MPATS) for university students (Xingtong and Chao, 2016).
4. Screening using the Self-Rating Anxiety Scale (SAS) to remove scores > 50 (patients with severe anxiety) (Jingsong et al., 2016).
5. Excluded students with less than a moderate degree of smartphone addiction tendency (mean score of 42.38) (Ganfang, 2017).
6. Excluded were students with mobile phone dependence scores below 60 (Lirong, 2015).
7. Exclude students with a score of 4 or below on the SAS-C (Kai, 2016).
8. Excluded smartphone addiction scores ≤ 65 and self-reported smartphone use ≤ 2 h/day were determined (Lan et al., 2018).
9. Exclude non-internet dependent persons with a score of 4 or below (Weifang et al., 2007).
10. Excluded students who scored < 3 on the Smartphone Addiction Scale (Yuxia et al., 2021).
11. Excluded students with sports contraindications and time conflicts (Renkai et al., 2015).
12. Excluded students with mental diseases, physical disabilities, or those who were unable or unwilling to participate in the trial (Kai, 2016).
13. Records of extreme physical or psychological problems, which includes different addictive disorders, psychotic disorders, primary depression, borderline personality disorder, or antisocial character disease primarily based on the clinical psychologist's view or observations and oral questioning (Alavi et al., 2021).
14. Excluded were students who had previously participated in cognitive group therapy sessions. Those students who had reported using medication to treat their mental disorders and who were receiving other psychotherapy were also excluded from the study (Alavi et al., 2021).
15. Those who have difficulty moving due to injury or illness, as well as those who are suspended or dropped out of school (Rui et al., 2018).
16. Inability to participate in exercise training independently (Lu et al., 2020).
17. They have a history of serious disease (e.g., cardiovascular disease, cerebrovascular disease, mental illness) or alcohol abuse (Lu et al., 2020).
18. They have participated with exercise in the past 3 months (e.g., walking, running, weight training, etc.) (Lu et al., 2020).

Sixth trials did not provide the exclusion criteria (Yu and Fumin, 2007; Wenhai and Jiamei, 2009; Wei et al., 2010; Ming et al., 2011; Li et al., 2017a; Zaihua et al., 2019).

#### Intervention

The most frequent exercise interventions included typical aerobic exercises such as Basketball + Badminton (Lirong, 2015; Rongchang and Xiaoyang, 2015; Kai, 2016; Xingtong and Chao, 2016; Xiaoni et al., 2019), volleyball (Renkai et al., 2015; Kai, 2016; Xingtong and Chao, 2016), Running (Jingsong et al., 2016; Ganfang, 2017), Tennis (Rongchang and Xiaoyang, 2015; Kai, 2016; Ganfang, 2017; Xiaoni et al., 2019), Cycling (Lirong, 2015; Fan et al., 2021), Football (Rongchang and Xiaoyang, 2015; Xiaoni et al., 2019), and Taijiquan + Yoga + Run + Badminton + Tennis (Ganfang, 2017). In addition, the most frequent psychological interventions were Group Counseling (GC) (Yu and Fumin, 2007; Wenhai and Jiamei, 2009; Wei et al., 2010; Zhang X. et al., 2020), Group Psychotherapy (GP) (Weifang et al., 2007), Mindfulness Cognitive-Behavioral Group Therapy (MCBGT) (Li et al., 2017a), Mindfulness Cognitive Therapy (MCT) (Rui et al., 2018), Group Mindfulness-based Cognitive-Behavioral Intervention (GMCI) (Lan et al., 2018), and Cognitive-Behavioral Group Therapy (CBGT) (Alavi et al., 2021).

Almost all exercise interventions were composed of 8–12 weeks, 2–5 sessions per week, with a duration of 40–90 min per session. All the sessions were completed by the students and the principal behavioral therapist, and they were done in a group format. Two studies demonstrated varying characteristics. First, Renkai et al. (2015) considered exercise training for 18 weeks, with 2 h (120-min) per session. Second, Fan et al. (2021) implemented acute aerobic cycling exercise intervention, and the exercise time was only 30 min, without reporting duration and frequency. Almost all psychological interventions were composed of 4–8 weeks, 1–2 weekly sessions, with a duration of 45 min−3 h per session. All the sessions were completed by the students and the principal behavioral therapist (Alavi et al., 2021). All the sessions were carried out by the researchers themselves (Ming et al., 2011) and teachers from psychological counseling centers (clinical psychological consultant) (Rui et al., 2018; Zaihua et al., 2019), and Master of Applied Psychology (Yu and Fumin, 2007). The study of one psychological intervention showed different characteristics. However, Alavi et al. (2021) implemented motor skill training as cognitive-behavioral group therapy, and its duration was 15 weeks.

Comparative Intervention was randomly divided into three groups and was composed of 12 weeks, two weekly sessions, and each ME (Qigong exercise) session (Lu et al., 2020) and GBT (cognitive behavior therapy) session lasted 90 min (Yuxia et al., 2021). All the sessions were completed by a certified coach-certified therapist (Lu et al., 2020).

The combined intervention was randomly divided into three groups and was composed of 10 weeks, two weekly sessions, with a duration of 60 min (moderate intensity aerobic exercise) per session (Yuxia et al., 2021). Heart rate = maximum heart rate × 70%; maximum heart rate = 220 – age. Heart rate variability for moderate load intensity ranged from 130 to 170 beats/min, and had a duration of 2 h (group psychological counseling) (Yuxia et al., 2021).

#### Comparisons

The most frequently applied control group in the studies considered was Usual Care (UC), or did not administer any treatment (Weifang et al., 2007; Yu and Fumin, 2007; Wenhai and Jiamei, 2009; Ming et al., 2011; Lirong, 2015; Renkai et al., 2015; Rongchang and Xiaoyang, 2015; Jingsong et al., 2016; Kai, 2016; Xingtong and Chao, 2016; Ganfang, 2017; Li et al., 2017a; Lan et al., 2018; Xiaoni et al., 2019; Zaihua et al., 2019; Lu et al., 2020; Zhang X. et al., 2020; Alavi et al., 2021; Fan et al., 2021; Xiao et al., 2021). However, several trials showed other or different control groups. Two studies focused on routine ideological and political education (Wei et al., 2010), and general health education (Rui et al., 2018). Furthermore, one study (Lu et al., 2020) compared mind-body exercise (i.e., ME), cognitive behavior therapy (i.e., CBT), and the control group. Another study (Yuxia et al., 2021) compared AE (Aerobic Exercise) with GPC (Group psychological counseling) and AE+GPC.

#### Outcomes

##### Primary outcomes

In most studies, there are four aspects of the primary outcome for assessed exercise interventions for smartphone addiction (withdrawal symptoms, highlight behavior, social comfort, mood change). The primary measurements used were Mobile Phone Addiction Index in Chinese (MPAI) (Lirong, 2015; Renkai et al., 2015; Xiaoni et al., 2019; Xiao et al., 2021), Mobile Phone Addiction Tendency Scale for College Students (MPATS) (Rongchang and Xiaoyang, 2015; Jingsong et al., 2016; Xingtong and Chao, 2016; Ganfang, 2017; Fan et al., 2021), and Smartphone Addiction Scale for College students (SAS-C) (Kai, 2016; Yuxia et al., 2021). Xiao et al. (2021) evaluated the outcome of addictive behavior: inability to withdrawal symptoms, control cravings, feeling lost and anxiety, loneliness, perceived stress, and productivity loss. In addition, measured heart rate (HR), reaction time (RT), and accuracy for exploring aerobic exercise can effectively have changes in the response inhibition in students that have smartphone addiction (Fan et al., 2021).

The primary measurement used Chinese Internet Addiction Scale (CIAS) (Yu and Fumin, 2007; Zhang X. et al., 2020), Young's Internet Addiction Questionnaire (YDQ), Symptom Checklist-90-Revised (SCL-90-R) (Alavi et al., 2021), Visual Analog Scale (VAS) (Yuxia et al., 2021), Self-Esteem Questionnaire (SES) (Wenhai and Jiamei, 2009), Emotional versus Social Loneliness (ESLS) (Wenhai and Jiamei, 2009; Ming et al., 2011), Pittsburgh Sleep Quality Index scale (PSQI) (Xiaoni et al., 2019). Cognitive Emotion Regulation (CERQ- C) (Wenhai and Jiamei, 2009), Social Avoidance and Distress (SAD) (Ming et al., 2011), and Wellbeing (Ming et al., 2011). In another study (Alavi et al., 2021), quality of life (QOL) was the main outcome. Lastly, Lu et al. (2020) investigated whether the addition of ME and CBT group protocol decreased anxiety, loneliness, perceived stress for a study population with addiction. And Yuxia et al. (2021) evaluated craving, Hamilton Depression Scale (HAMD) and Hamilton Anxiety Scale (HAMA).

##### Secondary outcomes

Mental health indices for anxiety [Self-Rating Anxiety Scale (SRAS)] (Lu et al., 2020; Xiao et al., 2021), loneliness [UCLA Loneliness Scale (UCLA-LS)] (Xiao et al., 2021), inadequacy [Field's Feelings of Inadequacy Scale (FIS) (Xiao et al., 2021), and stress (Chinese version of Perceived Stress Scale (CPSS)] (Xiao et al., 2021). ULS-8 Loneliness Scale (Lu et al., 2020), Perceived Stress Scale (PSS-14) (Lu et al., 2020).

These included feelings of inadequacy (FIS) and interference control (Flanker task). The timing of the measures of the outcome was variable, and it included assessment on a weekly basis for evaluation post-treatment. It also included 2, 3, 6, 14, and 20-month evaluations. However, seventeen works did not mention follow-up times (Yu and Fumin, 2007; Wenhai and Jiamei, 2009; Wei et al., 2010; Ming et al., 2011; Lirong, 2015; Renkai et al., 2015; Rongchang and Xiaoyang, 2015; Jingsong et al., 2016; Kai, 2016; Xingtong and Chao, 2016; Ganfang, 2017; Li et al., 2017a; Rui et al., 2018; Xiaoni et al., 2019; Zaihua et al., 2019; Lu et al., 2020; Fan et al., 2021). A review of mental fatigue-inducing interventions are shown in Tables 2–4.

**Table 2:** Overview of exercise intervention with smartphone addiction.

**Reference**	**Location**	**Participant characteristics**				**Intervention program**	**Motor skill training**			**Outcome** **measured**	**follow-up**
		**Sample size**	**Smartphone addiction level**	**Mean age or age range**	**Gender**		**Frequency (weekly)**	**Time (min)**	**Duration (week)**		
Renkai et al. (2015)	Nanchang, China	*n* = 36 (EG:18, CG:18)	Severe level	20.13 ± 1.35	M & F	EG: Volleyball CG: UC	3	120	18	MPAI ↑ (WS ↑, HB uncontrolled ↑)	NR
Lirong (2015)	Zhengzhou, China	*n* = 38 (EG: 20, CG: 18)	Severe level	20.33 ± 1.64 (freshman)	M & F	EG: Bicycle + Basketball + Badminton CG: UC	3	60	12	MPAI ↑ (WS ↑, HB uncontrolle ↑)	NR
Xingtong and Chao (2016)	Shandong, China	*n* = 49	Mild-to-moderate level	19.7 ± 1. 5	M & F	Basketball + Badminton +Run +Volleyball	3	90	10	MPATS ↑ (WS ↑; SC ↑; MC ↑; HBsalience ↑)	NR
Rongchang and Xiaoyang (2015)	Nanjing, China	*n* = 754 (EG: 344, CG: 410)	NR	18–22 (freshman)	M & F	EG: Basketball + Badminton + Football + Tennis CG: UC	5	45–60	12	MPATS ↑ (WS ↑; SC↑; MC ↑; HB salience ↑)	NR
Kai (2016)	Taiyuan, China	*n* = 73 (EG: 36, CG: 37)	Mild-to-moderate level	18–22	M & F	EG: Basketball +Table tennis + Badminton + Volleyball CG: UC	3	45	12	SAS-C ↑ (WS ↑; SC ↑; MC ↑; HB salience ↑)	NR
Jingsong et al. (2016)	Hunan, China	*n* = 80 (EG: 40, CG: 40)	Mild-to-moderate level	18–22	M & F	EG: Run CG: UC	2	45	8	MPATS ↑ SRAS (WS ↑; SC ↑; MC ↑; HB salience ↑)	NR
Ganfang (2017)	Zhejiang, China	*n* = 60 (EG: 30, CG: 30)	Mild-to-moderate level	20.72 ± 1.30	M & F	EG: Taijiquan + Yoga + Run + Badminton + Tennis CG: UC	3	60	8	MPATS↑ (WS ↑; SC ↑; MC ↑; HB salience ↑)	NR
Xiaoni et al. (2019)	Hunan, China	*n* = 99 (EG: 50, CG: 49)	Mild-to-moderate level	18–20	F	EG: Basketball + Badminton + Football + Tennis CG: UC	4	60	8	MPAI ↑ PSQI ↑	NR
Xiao et al. (2021)	Central China	*n* = 100 (EG1: 33 EG2: 33 CG:34)	Mild-to-moderate level	Baduanjin:19.21 ± 1.02. Basketball: 18.95 ± 0.89; Control:19.71 ± 1.7	M & F	EG1: Basketball; EG2: Baduanjin; CG: UC	3	90	12	MPAI ↑ SRAS ↑; UCLA-LS ↑; FIS ↑ PSS-14 ↔	2 months
Fan et al. (2021)	NR	*n* = 30 (study1: 15; Study2: 15)	Mild-to-moderate level	study 1: 20.03 ± 0.96; Study 2 :19.87 ± 0.99	M & F	EG: Acute aerobic cycling exercise. CG: UC	NR	30	NR	MPATS ↑ Go/NoGo task;; RT ↑; Ac ↑; HR; Flanker task ↑	NR

M, Male; F=Female; EG, experimental group; CG, control group; UC, Usual Care; MPAI, smartphone addiction index; MPATS, Mobile phone addiction tendency scale; WS, withdrawal symptoms; HB, highlight behavior (include: inability to control craving, withdrawal and escape); SC, social comfort; MC, mood change; SAS-C, Smartphone Addiction Scale for College students; PSQI, Pittsburgh Sleep Quality Index scale; SRAS, Self-Rating Anxiety Scale; UCLA-LS, UCLA Loneliness Scale; FIS, Field's Feelings of Inadequacy Scale; PSS-14, Perceived Stress Scale; RT, Reaction Time; Ac, accuracy; HR, heart rate; NR, not reported. Smart phone addiction level: 40–60 points = mild-to-moderate level; more than 60 points = severe level. Highlight behavior: uncontrolled and salience are emphasizing the importance of using mobile phone on individuals, so we merged them into one item of highlight behavior. ↑, significant difference with-group from pretest-posttest; ↔, no significant difference.

**Table 3:** Overview of psychosocial intervention with smartphone addiction.

**Reference**	**Location**	**Participant characteristics**				**Intervention program**	**Motor skill training**			**Outcome** **measured**	**follow-up**
		**Sample size**	**Smartphone addiction level**	**Mean age or age range**	**Gender**		**Frequency (weekly)**	**Time (min/hour)**	**Duration (week/ sessions)**		
Yu and Fumin (2007)	Beijing, China	*n* = 48 (EG: 24, CG: 24)	Mild-to-moderate level	19 ± 2	M & F	EG: Group Counseling CG: No treatment	2	2 h	4 weeks	CIAS ↑ SCL – 90 ↔ IA-Sym (Sym -C; Sym -W; Sym -T); IA-RP (RP-IH; RP-TM)	NR
Weifang et al. (2007)	Zhejiang, China	*n* = 61 (EG: 30, CG: 31)	Mild-to-moderate level	21.8 ± 1.2	M & F	EG: Group psychotherapy; CG: No treatment	1	50-min	8 weeks	YDQ ↑ SCL – 90 ↑	3 & 6 months
Wenhai and Jiamei (2009)	Jiangsu,China	*n* = 37 (EG: 12, CG1: 13, CG2:12)	NR	17–21	M & F	EG: Group Counseling CG: No treatment	1	3 h	8 sessions 8 weeks	YDQ ↑ SES ↑; ESLS ↑; CERQ- C ↑	NR
Wei et al. (2010)	Jiangsu, China	*n* = 160 (EG: 80, CG:80)	Mild-to-moderate level	21 ± 1	M & F	EG: Centralized and Closed Group Counseling therapy CG: Political thoughts course	1	5 h	4 weeks	YDQ ↑ (WS ↑; TM ↔; RA ↔)	NR
Ming et al. (2011)	Suzhou, China	*n* = 71 (EG: 36, CG: 35)	NR	Not reported	M & F	EG: Group Guidance CG: No treatment	1	2 h	8 weeks	IAT ↑ MC ↑; SAD ↑; IWB ↑; ESLS ↑;	NR
Li et al. (2017a)	Jinzhou, China	*n* =20 (EG:10; CG:10)	NR	19.2 ± 1.1	M & F	EG: Mindfulness Cognitive-Behavioral Group Therapy CG: No treatment	1	2.5 h	8 weeks	SAS ↑ MA ↑; BIS-11 ↑; SRAS ↑	NR
Rui et al. (2018)	Zhengzhou, China	*n* = 82 (EG: 41, CG: 41)	NR	17–23	M & F	EG: Mindfulness cognitive therapy CG: Health education	NR	45-min	7 sessions 4 weeks	MPATS ↑; IAT ↑ (WS ↑; SC ↑; MC ↔; HB salience ↑; IH ↑)	NR
Lan et al. (2018)	Shanghai, China	*n* = 70 (EG: 41, CG: 29)	Severe level	21.3 ± 1.3	M & F	EG: Group mindfulness-based cognitive-behavioral intervention CG: No treatment	1	1 h	8 weeks	MPIAS ↑ SUT ↔ T1↔; T2 ↑; T3 ↑; T4 ↑	14th and 20th week
Zaihua et al. (2019)	Hunan, China	*n* = 68 (EG: 34, CG: 34)	NR	Not reported	M & F	EG: Cognitive-behavioral interactive group therapy CG: No treatment	1	NR	8 weeks	MPATS ↑ (WS; SC; MC; HB salience)	NR
Zhang X. et al. (2020)	Chongqing, China	*n* = 18 (EG: 9, CG: 9)	Moderate-to- high levels	EG: 20.11 ± 1.45 CG: 20 ± 1.56	M & F	EG: Group Counseling Intervention CG: No treatment	1	2.5 h	5 weeks	CIAS-R ↑ IA-Sym ↑ (Sym-C & Sym-W ↑); IA-RP ↑ (Sym-T ↑; RP-IH ↑; RP-TM ↑); SCL-90	6-month
Alavi et al. (2021)	Tehran, Iran	*n* = 50 (EG: 25, CG: 25)	NR	18–30	M & F	EG: Cognitive-behavioral group therapy CG: No treatment	1	90-min	15 sessions 15 weeks	IAT ↑; QOL ↑; MH ↑; SCL-90-R ↑ Semi-structured interview	3-month

IH, Interpersonal and Health; NE, negative effect; CIAS, Chinese Internet Addiction Scale; SCL-90, Symptom Checklist-90; SCL-90-R, Symptom Checklist-90-Revised; IA-Sym, Internet Addiction Core Symptoms; IA-RP, Internet Addiction Related Problem; Sym -C, Compulsive Symptoms of Internet Addiction; Sym-W, Withdrawal symptoms of Internet Addiction; Sym- T, Tolerance Symptoms of Internet Addiction; RP-IH, Interpersonal and Health-Related Problems of Internet Addiction; RP-TM, Time Management Problems; RA, Real alternative; IAT, Internet addiction test; YDQ, Young's Internet Addiction Questionnaire; SES, Self-Esteem Ques-tionnaire; ESLS, Emotional versus Social Loneliness Scales; MA, mental awareness; BIS-11, Barratt Impulsivity Scale; SRAS, Self-Rating Anxiety Scale; CERQ-C, Cognitive Emotion Regulation Questionnaire; SAD, Social Avoid-ance and Distress Scale; CIAS-R, Chinese Internet Addiction Scale; IWB, Index of Wellbeing; QOL, Quality of Life; MH, Mental Health; MPATS, Mobile phone addiction tendency scale; SUT, Smartphone use time; T1, the baseline measurement (1st week); T2, the post-intervention (8th week); T3, the first follow-up (14th week); T4, the second follow-up (20th week).

‡, significant difference with-group from pretest-posttest; ↔, no significant difference.

**Table 4:** Overview of combined intervention with smartphone addiction.

**References**	**Location**	**Participant characteristics**				**Intervention program**	**Motor skill training**			**Outcome measured**	**Follow-up**
		**Sample size**	**Smartphone addiction level**	**Mean age or age range**	**Gender**		**Frequency (weekly)**	**Time (min/ hour)**	**Duration (week/sessions)**		
Lu et al. (2020)	Central China	*n* =95 (EG1:34 EG2:34 CG:34)	Mild-to-moderate level	19.23	M &F	EG1:ME EG2: CBT CG: Usual Care	2	90-min	12	MPAI ↑ SRAS ↑; ULS-8 ↑; PSS-14↓	NR
Yuxia et al. (2021)	Henan, China	*n* =148 (EG1: 49 EG2: :50 CG: 49)	Mild-to-moderate level	EG1:20. 21 ± 1. 19 EG2:19. 81 ± 1. 21 CG: 20. 14 ± 1. 27	M & F	EG1: Aerobic exercise EG2: Group psychological counseling CG: Aerobic exercise + Group psychological counseling	EG1: 2 EG2: 1	EG1: 60-min; EG2: 2 h	(1) EG1:10 weeks (2) EG2: 10 sessions	SAS-C ↑; VAS ↑; HAMD ↑; HAMA ↑	3-month

SRAS, Self-Rating Anxiety Scale; ULS-8, using the ULS-8 Loneliness Scale; PSS-14, Perceived Stress Scale; SAS-C, Smartphone Addiction Scale; VAS, Visual Analog Scale; HAMD, Hamilton Depression Scale; HAMA, Hamilton Anxiety Scale. ↑, significant difference with-group from pretest-posttest; ↓, significantly decreased (However, no significant difference with-group from pretest-posttest).

##### Synthesis of results

The results after exercise intervention showed that there was a significant difference (*P* < 0.01) between the experimental group and control group in smartphone addiction, and the detection rate of smartphone addiction was 21.6 and 39.6%, respectively, with a significant difference (*P* < 0.05); there was a significant difference between the experimental group and the control group in the PSQI score (*P* < 0.01), and the detection rate of sleep problems was 11.8 and 29.2%, respectively, with a significant difference (*P* < 0.05). The difference was significant (*P* < 0.05) (Xiaoni et al., 2019). Exercise reduced smartphone addiction (MPATS score) (Lan et al., 2018; Xiao et al., 2021), and withdrawal symptoms, highlight behavior, social comfort, mood change (*p* < 0.01) (Rongchang and Xiaoyang, 2015; Ganfang, 2017).

Mobile phone addiction tendency total score of between group (experimental group and control group), within group (experimental time), and interaction effect (*P* < 0.05), Physical exercise reduced the effect values of smartphone addiction and four dimensions in university students, and their behavior change had a significant improvement effect (Ganfang, 2017).

Self-Esteem Questionnaire (SES) (*p* < 0.01) (Wenhai and Jiamei, 2009), Emotional vs. Social Loneliness (ESLS *p* < 0.01) (Wenhai and Jiamei, 2009; Ming et al., 2011), Cognitive Emotion Regulation (CERQ- C, *p* < 0.01) (Wenhai and Jiamei, 2009).

Basketball and Baduanjin have a significant effect on the reduction of smartphone addiction (*p* < 0.01), and mental health (such as anxiety, loneliness, inadequacy, and stress (basketball: *p* < 0.01; Baduanjin: *p* = 0.04). After the 2-month follow-up, both exercise interventions have significant effects on reduced smartphone addiction, and improve mental health.

Duration of use smartphone in experimental group was significantly lower than the control group and the score of MPAI (*P* < 0.01). The inability to control craving, withdrawal and escape (*P* < 0.05). Productivity loss were significantly lower than the control group when after exercise intervention (Renkai et al., 2015).

Aerobic sport has significant effect on the reduction of smartphone addiction (MPAI, *p* < 0.01) (Lirong, 2015). Moderate intensity had the greatest effect on inhibitory control of smartphone addiction. NoGo stimulus (*p* = 0.012), and the RT of Go stimulus (*p* ≤ 0.001) (Fan et al., 2021).

After the 12-week exercise intervention, the smartphone addiction scale scores of university students in the experimental group decreased significantly (*P* < 0.01) compared to the control group, and the decrease was more pronounced in male students than in female students (*P* < 0.05) (Kai, 2016).

There was an interaction effect of intervention and time on total IAT and MPATS scores (*P* < 0.001), with significant differences between the two groups in tolerance and smartphone usage time control, interpersonal relationships and health, withdrawal response and social comfort (*P* < 0.05) (Rui et al., 2018).

The cognitive-behavioral group therapy (CBGT) showed reduction in scores of internet addiction, quality of life (QOL) and mental illness (*p* < 0.05) in university students with Internet addiction (Alavi et al., 2021). loneliness, anxiety (*p* < 0.001 for ME vs. CG) (Lu et al., 2020).

After combining with group psychological training intervention and 3 months after the intervention, compared with the pre-intervention period, the SAS-C, VAS, HAMD, and HAMA scores of the 3 groups tended to decrease with time (*P* < 0.01), and the scores at the same time points were the lowest in the exercise and group counseling, the second highest in the group counseling group, and the highest in the exercise group (*P* < 0.01). The lowest scores were in the exercise + group counseling, followed by the group counseling, and the highest scores were in the exercise group (*P* < 0.01). Three months after the intervention, the subjects in the three groups still had depression and anxiety symptoms (Yuxia et al., 2021).

## Discussion

In the review, we focus on the basic areas of exercise and psychological intervention for smartphone addiction: study selection and design, study characteristics (participants, intervention, comparisons, and outcomes).

The target groups were university students. Given the current prevalence of most smartphone addiction among university students (Sunday et al., 2021), it is critical to focus on this particular group. There are studies on exercise interventions for smartphone addiction and studies related to psychological interventions for smartphone addiction, but there are few or no studies on the combination of exercise and psychological interventions for smartphone addiction. Previous studies have mentioned that combining exercise and psychological interventions may be more beneficial in reducing smartphone addiction, and the results of this study also confirmed the hypothesis of this study. In order to address the impact of smartphone addiction on university students' mental and physical health, future interventions are better focused on combining interventions.

Targeting the smartphone addicted university student population can be achieved through a combination of exercise and psychological interventions. Although we can find several recommendations for exercise and psychological interventions for smartphone addiction in the literature, only one study (Yuxia et al., 2021) has investigated the impact of exercise and psychological interventions on smartphone addiction. Therefore, researchers should design and implement scientifically rigorous evaluations of studies combining exercise and psychological interventions for smartphone addiction.

Nevertheless, in most of the included trials, only one article, where the effects persist at follow-up assessment, proved the lasting effect of exercising in the long run (Xiao et al., 2021).

The psychosocial intervention saw less smartphone usage time during post-intervention, and the first two follow-ups, as well as the lower MPIAS and YDQ scores at follow-up, proved the lasting effect of the mindfulness-based intervention (MBI) and group psychotherapy in the long run (Weifang et al., 2007; Lan et al., 2018).

In order to discuss the impact of combining exercise and psychological interventions on smartphone addiction, it is necessary to conduct more research on the effectiveness of exercise and psychological interventions in smartphone addiction.

### Efficacy of exercise intervention with smartphone addiction

Exercise increases university students' escape psychology, and the frequency of physical exercise sessions was substantially connected with anxiety and social relationships for university students. Furthermore, after the exercise intervention, the ratings for loss of control and low efficacy components were considerably less than in the control group.

Wang et al. found that an exercise intervention delivered solely to heavily smartphone dependent university students was insufficient (Xingtong and Chao, 2016). Medical students with severe mobile phone addiction should participate in co-therapies that include pharmacological and psychological interventions. Improvements in heavy mobile phone addiction symptoms will also require increased research efforts with proven measures.

The effect of exercise intervention for college students of different genders is slightly different for different measurement dimensions. The intervention effect of female students is better than that of male students in withdrawal symptoms and highlighting behavior dimensions. However, there was no significant difference in the total scale score between male and female students (Rongchang and Xiaoyang, 2015).

Kai (2016) found that there was a significant difference in the intervention effect of mobile phone addiction among students between genders, and the intervention effect of male students was better than that of female students, which was inconsistent with previous research results (Rongchang and Xiaoyang, 2015). There are many reasons for the inconsistent results, such as different measurement tools used, intervention time, preliminary tests, exercise intensity, and intervention plan. The results caused by intervention may be different. In later research on sports intervention for students' mobile phone addiction, we can try to improve the intervention effect by combining psychological intervention, drug intervention, and other comprehensive intervention methods, and explore the intervention effect and timeliness of different sports.

It was confirmed that Tai Ji Chuan, yoga, and jogging as exercise programs for withdrawal behaviors could alleviate symptoms such as anxiety, disturbance, palpitation, and accelerated heartbeat (Ganfang, 2017). Badminton, tennis, and running mood-changing exercise programs can change negative psychology. PSU students had more extensive upgrades in mental health by way of group-based basketball intervention as compared to Baduanjin intervention (Xiao et al., 2021).

Comprehensive exercise-based intervention (Xiaoni et al., 2019) has a significant effect on alleviating the symptoms of mobile phone reliance among university students and improving their sleep quality. The study has shown that mobile phone dependence positively correlates with sleep quality.

Moderate-intensity exercise enhances inhibitory control in university students who have a smartphone addiction (Fan et al., 2021). Based on the Strength Model of Self-Control, self-control depends on a restricted strength valuable resource (Baumeister et al., 2007). The arousal factor within the reticular activation model can be better activated by sports or exercise (Lambourne and Tomporowski, 2010; Dietrich and Audiffren, 2011).

### Efficacy of psychosocial intervention with smartphone addiction

Group psychological counseling can more effectively improve the emotional adjustment and expression ability of addiction and change the emotional state of students (Wenhai and Jiamei, 2009). Ming et al. suggest that group counseling has a positive effect on reducing social anxiety levels, establishing social support systems, and reducing internet-dependent behaviors.

Rui et al. (2018) established a stable and healthy social support system and enhanced individuals' self-esteem and identity. This study combined positive thinking and internal cognitive therapy characteristics, supplemented with a group therapy model, which led to partial improvement of the cell phone addiction problem among college students. The study method is easy to operate, low cost has no adverse effects, and can be further validated and promoted for use.

In many studies, MBIs have completed great consequences on some behavioral addictions, including pathological gambling (de Lisle et al., 2012), workaholism (Shonin et al., 2014b), sex addiction (van Gordon et al., 2016), and internet addiction (Shonin et al., 2014a; Lan et al., 2018). However, only a few MBI research works on smartphone addiction prevention have been conducted (Lan et al., 2018).

### Efficacy of combined intervention with smartphone addiction

One of the trials that compared ME and CBT reported that mindfulness (e.g., Qigong or Baduanjin) training had a significant advantage in the treatment of substance use compared to CBT and usual care (Sancho et al., 2018; Lu et al., 2020). Additionally, the results seen in this study are reasonably in agreement with those by Bowen et al. (2014), who show that drug addicts who engaged in mindfulness training or c for a 6 month period saw a decline in drug usage. However, mindfulness training had a higher decrease in this outcome compared to CBT at a 1-year follow-up duration (Bowen et al., 2014; Lu et al., 2020). The results reported in this work show that both ME and CBT can be impactful in decreasing social problems and enhancing good mental health (i.e., reduced loneliness, stress and anxiety) for university student smartphone addiction (Lu et al., 2020).

The results of this study show that exercise, group counseling, and combined exercise and group counseling can suppress the psychological craving and addiction and the co-morbid depression and anxiety of smartphone addicts to different degrees. Combined exercise and group counseling are more significant than the other two groups. The physical strengthening through exercise participation would positively impact the cognition, mood, and behavior of the intervention subjects, which in turn enhances mental health. Exercise intervention (exceptionally moderate-intensity exercise) has shown good improvement in the prevention and treatment of internet addiction (de Souza Cortes et al., 2002; Ramos-Jorge et al., 2014; Yuxia et al., 2021). The organic combination of exercise therapy and group counseling, both ideal low-cost interventions, has some value for dissemination. However, there is a lack of research on the synergistic benefits between multiple interventions.

Overall, in the above study of exercise and psychological interventions for smartphone addiction, the authors found the effect of combined exercise and group psychological counseling to be more significant than that of the other two groups. However, the subjects still had depression and anxiety symptoms after the follow-up visit, indicating that the intervention plan still needed further exploration and adjustment, or it needed to be combined with other intervention methods to improve the intervention effect (Yuxia et al., 2021). Additionally, these works tend to show that a combination of psychological interventions and exercise would be the optimal treatment option. Combining exercise and psychological interventions is an effective readily accessible and low-cost training regimen with a particular promotion value (Lu et al., 2020).

Very few countries have implemented a combination of exercise and psychological interventions in practice. No efficacy or effectiveness studies have been conducted. We encourage researchers and students treating smartphone addiction/internet addiction to implement and study combined interventions.

The advantage of this review is that (to the authors' knowledge), it is the first review to focus on exercise and psychological interventions for smartphone addiction, which also includes text written not only in English, but also in Chinese. Several limitations are worth noting. First, the majority of the sample sizes were small. Second, most studies did not control the confounders.

The 23 literature gives support to the effectiveness of the exercise and psychological interventions, which includes one study showing comparative effectiveness of mind-body exercise vs. cognitive behavioral may effectively reduce the level of smartphone addiction. A few studies have shown that combined exercise and psychological interventions are more combined effects in suppression compared to single psychological intervention and exercise intervention groups. However, there is a lack of additional studies to validate the effectiveness of combined interventions.

In most of the exercise intervention studies were ball sports (i.e., basketball and badminton), it is suggested that in future studies, exercise interventions might be more inclusive of aerobic exercises besides ball sports. Recently mindfulness-based interventions (MBI) have been widely used in behavioral addiction research.

There was one study which showed that a mindfulness intervention was significant to reduce smartphone addiction among severe addicted university students (score ≥ 65) (Lan et al., 2018). However, there are few evidence-based studies of behavioral addiction using exercise and MBI.

Through the duration of previous studies for exercise and psychological interventions, we found that 9 out of 23 studies were conducted in 8 weeks. Among the outcome measures of the smartphone addiction studies found to be insufficient research on inhibitory control. in the current study of smartphone addiction among university students has only one study focused on female university students with smart addiction.

## Conclusion and future perspectives

Prior work in the literature promotes the success of psychosocial interventions and exercise. These treatments are sufficient to decrease dependence, cravings, as well as related addiction symptoms, and to enhance mood state and emotion problems. Particular interventions showed better outcomes for the treatment of smartphone addiction, including CBT, GMCI, CBGT, MBI, MBIs, or MCBGT. Nevertheless, the best effects may be the combination of exercise and psychosocial intervention or a different active treatment. Only a handful of works found maintenance of the impact over time, and it would be crucial to perform more further studies in the future. Previous work has shown that moderate-intensity exercises had the best impact on response inhibition. Aerobic exercise is highly beneficial to promote inhibitory control for university students who suffer from smartphone addiction, and these students can have major inhibitory control deficits (Chen et al., 2016; Moisala et al., 2016; Gao et al., 2020; Fan et al., 2021). However, there no studies are available on the impact of combining both exercise and psychological intervention on the inhibitory control, and executive and cognitive function, of smartphone addiction.

Two state-of-the-art models of internet gaming disorder or internet addiction were proposed in the last few years (Young and Brand, 2017). Dong and Potenza's (2014) model concentrates on the cognitive-behavioral functionality of internet gaming disorder and offers treatment recommendations and various treatment strategies. It provides a model that explains internet gaming disorder includes cognitive components, decision-making styles, as well as motivational components, which are resolved by a series of therapeutic approaches (Dong and Potenza, 2014; Young and Brand, 2017).

As for the target population, females are more probable to become addicted to smartphones compared to males (Demirci et al., 2015; Gutiérrez et al., 2016; Sohn et al., 2019; Mehmood et al., 2021), and females are also more probable to have increased problematic use of smartphones (Takao et al., 2009; Kim et al., 2016). The previous studies reported that females were 1.4 times more inclined to smartphone addiction compared to males (Kim et al., 2016; Chen et al., 2017). Other recent studies also empirically prove that females are more addicted to smartphones compared to males (Kim et al., 2016; Chen et al., 2017; Busch and McCarthy, 2021; Yoon et al., 2021). However, there was no significant difference in smartphone addiction between men and women in some research (Yen et al., 2009; Dixit et al., 2010; Mehmood et al., 2021). Further empirical studies are encouraged to investigate addiction problems in females, because females are a fragile and sensitive population and more addicted to smartphones.

This systematic review found that a combination of exercise and psychological intervention was more effective in reducing smartphone addiction, and exercise and psychological interventions can be extended to other behavioral addictions. The proposed future should focus on university students and young female vulnerable to smartphone addiction or other addiction-related problems. Focus on the effects of exercise and psychological intervention on inhibitory control, cognitive function and executive function of university students' smartphone addiction.

## Limitations

The systematic review is reported to show the results and effects of exercise and psychological interventions. The main limitation of this review is the inclusion of only databases using English and Chinese languages, and this study finds most of the samples were from China, while there are still many relevant studies in other countries or regions. Currently smartphone addiction is increasing across the globe (Olson et al., 2022), it is recommended that more countries be involved in this study.

## Future directions

Some research additionally showed a positive relation of smartphone addiction and physiological health (Shoukat, 2019). However, currently most of the research is on the psychological aspects of smartphone addiction among university students, and few studies have been conducted from the physiological direction. There are physiological aspects focus on the effects of sleep quality. There is no research to focus the physiological direction of smartphone addiction (such as visual acuity, visual responsiveness). The psychological aspects lack research on the neurocognitive mechanisms, emotional, cognitive responses, and executive function aspects of smartphone addiction.

Furthermore, there is no research in the area of neuroscience, such as magnetic resonance imaging (MRI) (Liu et al., 2006; Singh, 2014), magnetoencephalography (MEG) (Liu et al., 2006; Singh, 2014), and electroencephalography (EEG) (Liu et al., 2006; Singh, 2014), functional magnetic resonance imaging (fMRI) (Liu et al., 2006) on the exercise and psychological interventions in the direction of smartphone addiction. And there is lack of research protocols on combined interventions in the physiological and psychological direction.

Finally, further studies should focus on the cross-section of neuropsychology, cognitive psychology, and sports science to provide viable interventions and scientific guidance for smartphone addiction among university students.

## Data availability statement

The original contributions presented in the study are included in the article/Supplementary material, further inquiries can be directed to the corresponding author/s.

## Author contributions

HL and FQ performed the selection of studies and search of the literature. HL did the primary screening of titles and abstracts, did the quality assessment of the study, interpreted the data, and wrote the manuscript. HL and KS individually reviewed all the considered abstracts and eligible articles using the predefined inclusion criteria. KS resolved any potential disagreements in the study inclusion. All authors contributed to the manuscript initiation, revision, read, and approved the final version.

## Conflict of interest

The authors declare that the research was conducted in the absence of any commercial or financial relationships that could be construed as a potential conflict of interest.

## Publisher's note

All claims expressed in this article are solely those of the authors and do not necessarily represent those of their affiliated organizations, or those of the publisher, the editors and the reviewers. Any product that may be evaluated in this article, or claim that may be made by its manufacturer, is not guaranteed or endorsed by the publisher.
